The article "EGFR, FLT1 and Heparanase as Markers Identifying Patients at Risk of Short Survival in Cholangiocarcinoma" was published in 2013. Journal: PLoS One.

# EGFR, FLT1 and Heparanase as Markers Identifying Patients at Risk of Short Survival in Cholangiocarcinoma

**DOI:** 10.1371/journal.pone.0064186

**Published:** 2013-05-21

**Authors:** Andreas-Claudius Hoffmann, Eray Goekkurt, Peter V. Danenberg, Sylvia Lehmann, Gerhard Ehninger, Daniela E. Aust, Jan Stoehlmacher-Williams

**Affiliations:** 1 Department of Medical Oncology, West German Cancer Center, University Duisburg-Essen, Essen, Germany; 2 Department of Oncology, Hematology and Stem Cell Transplantation, University Hospital Aachen, RWTH University Aachen, Aachen, Germany; 3 Department of Biochemistry and Molecular Biology, and Norris Comprehensive Cancer Center, University of Southern California, Los Angeles, California, United States of America; 4 Internal Medicine Clinic I, Carl Gustav Carus University Hospital, Dresden, Germany; 5 Institute of Pathology, Carl Gustav Carus University Hospital, Dresden, Germany; University of Connecticut Health Center, United States of America

## Abstract

**Background:**

Cholangiocarcinoma remains to be a tumor with very few treatment choices and limited prognosis. In this study, we sought to determine the prognostic role of fms-related tyrosine kinase 1/vascular endothelial growth factor receptor 1 (*FLT1/VEGFR1*), heparanase (*HPSE*) and epidermal growth factor receptor (*EGFR*) gene expression in patients with resected CCC.

**Methods:**

47 formalin-fixed paraffin embedded FFPE tumor samples from patients with resected CCC were analyzed. FFPE tissues were dissected using laser-captured microdissection and analyzed for *FLT1*, *FLT4*, *HPSE*, *Hif1a*, *VEGFA/C*, *HB-EGF*, *PDGFA*, *PDGF-RA and EGFR* mRNA expression using a quantitative real-time RT-PCR method. Gene expression values (relative mRNA levels) are expressed as ratios between the target gene and internal reference genes (beta-actin, b2mg, rplp2, sdha).

**Results:**

*EGFR*, *FLT1* and *HPSE* expression levels were significantly associated with overall survival (OS). *FLT1* showed the strongest significant independent association with overall survival in a multivariate cox regression analysis when compared to the other genes and clinicopathological factors with a nearly 5 times higher relative risk (4.74) of dying earlier when expressed in low levels (p = 0.04). ROC Curve Analysis revealed that measuring *EGFR* potentially identifies patients at risk of a worsened outcome with a sensitivity of 80% and a specificity of 75% (p = 0.01).

**Conclusions:**

*EGFR* and *FLT1* seem to be potential markers to identify those patients at high risk of dying from cholangiocarcinoma. Therefore these markers may help to identify patient subgroups in need for a more aggressive approach in a disease that is in desperate need for new approaches.

## Introduction

The treatment of solid tumors has seen a lot of progress over the last few years with significant survival benefits in diseases like breast and colorectal cancer especially through the development of several new molecular entities. Nonetheless in cholangiocarcinoma respectively cancers of the biliary tract the treatment choices remain very limited [1], [2]. Cholangiocarcinoma seems to be a cancer with an inhomogeneous genetic design influenced by multiple molecular aberrations limiting the successful application of conservative approaches to find new treatments by simply adding new molecular entities (NME, i.e. small molecules) to classical cytotoxic regimes [3]. Identifying patient subgroups with more aggressive subtypes of CCC at risk for a shortened survival may lead to improved trial designs and hence to a more effective strategy in treating this disease.

By previous work we already identified several candidate biomarkers that are associated with the overall survival of patients in various cancer types. These genes have a strong correlation with angiogenesis (*Hif1a*, *FLT1*) [4], [5] and lead to alterations of the extracellular matrix and remodeling of subepithelial and subendothelial basal membranes (heparanase, *HPSE*) [6], [7] and therefore seem to be directly involved in the aggressiveness of cancers.

In this study, we investigated the prognostic values of fms-related tyrosine kinase 1/vascular endothelial growth factor receptor 1 (*FLT1/VEGFR1*), heparanase (*HPSE*), hypoxia inducible factor 1, alpha subunit (*Hif1a*), fms-related tyrosine kinase 4/vascular endothelial growth factor receptor 3 (*FLT4/VEGFR3*), vascular endothelial growth factor A & C (*VEGFA/C*), platelet-derived growth factor alpha polypeptide A (*PDGFA*), PDGF receptor, alpha polypeptide (*PDGF-RA*) heparin-binding EGF-like growth factor (*HB-EGF*), and epidermal growth factor receptor (*EGFR*) gene expressions as well as their interrelationships in cholangiocarcinoma. We measured the mRNA expression levels of these genes with quantitative real-time reverse transcriptase-PCR (RT-PCR) in laser-microdissected formalin-fixed paraffin-embedded (FFPE) tissue samples of cholangiocarcinoma. This approach was taken to get a more precise result of gene expression than previously available since stromal tissue might significantly influence results and identification of significant genes [8]. We then further analyzed the abovementioned genes and their correlation with clinical and histopathological variables such as primary tumor stage (pT, based on the International Union Against Cancer, UICC, 1997), regional lymph node metastasis, grading and overall survival.

## Materials and Methods

### Study Population and Tumor Samples

FFPE samples were obtained from patients with cholangiocarcinoma with a median age of 73 years (range 48–93 years) at time of diagnosis. All patients received gemcitabine-based chemotherapy and were treated at the University hospital of Dresden, Germany between 2001 and 2007. Patient demographics are listed in Table 1. TNM staging was performed according to the criteria of the International Union Against Cancer [9]. All samples where reviewed by a board certified clinical pathologist. Clinical diagnosis and staging was done according to local guidelines using among others endoscopy and CT-Scans. This study and the herein used retrospective genetic analysis was approved by the local ethics committee in Dresden, Germany. The Name of the ethics committee is “Ethikkommission der Medizinischen Fakultät, TU Dresden” (Fetscherstrasse 74, 01307 Dresden) and the Reference Number for the ethic statement is EK137072006. The requirement for patient consent was specifically waived by the approving IRB.

**Table 1:** Patient Characteristics.

Age	
median (range), years	74 (48–93)
Gender	
female	37 (78.7%)
male	10 (21.3%)
Primary tumor expansion (pT)	
pT1	6 (12.8%)
pT2	17 (36.2%)
pT3	20 (42.6%)
pT4	3 (6.4%)
Lymph node involvement (pN)	
pN0	37 (78.7%)
pN1	10 (21.3%)
Grade of Dedifferentiation (G)	
G2	17 (36.2%)
G3	28 (59.6%)
Overall Survival	
median (range), months	13 (0–69)

The clinico-pathological characteristics of all patients were reviewed by a surgical pathologist. Representative hematoxillin and eosin-stained slides of Formalin-fixed, paraffin-embedded (FFPE) tissue blocks obtained at cholecystectomy or from biopsies were reviewed in order to estimate the tumor load per sample. For laser-captured microdissection (P.A.L.M. Microlaser Technologies AG, Munich, Germany) slides of 10 µm thickness were obtained. All tumor slides were prepared as described previously [4].

### Quantitative Real-time Polymerase Chain Reaction

RNA was isolated from microdissected tumor samples following a proprietary procedure at Response Genetics Inc (Los Angeles, CA; US patent No. 6248,535). The resulting tumor RNA was reverse transcribed into cDNA as described previously [4]. Expression of *FLT1*, *FLT4*, *HPSE*, *Hif1a*, *VEGFA/C*, *HB-EGF*, *PDGFA*, *PDGF-RA*, *EGFR* and *internal reference genes (beta-actin, b2mg, rplp2, sdha) was* quantified by real-time fluorescence detection of amplified cDNA (ABI PRISM 7900 Sequence Detection System [TaqMan], Perkin-Elmer Applied Biosystems, Foster City, CA). The reverse transcription and polymerase chain reaction (RT-PCR) assay was implemented as described previously [4]. All primers were selected using the Gene Express software (Applied Biosystems, Foster City, CA), but were adapted to the requirements of cDNA generated from RNA, which was extracted from FFPE tissue. All primers were validated following a previously described protocol [5]. All genes were run on all samples in triplicates, i.e. one sample was run with each gene three times on the same plate to identify potential outliers. The detection of amplified cDNA results in a cycle threshold (Ct) value, which is reciprocal to the amount of cDNA contained in the sample. Normal colon, liver, and St. Universal Mix RNA (Stratagene, La Jolla, CA) were used as control calibrators on each assay plate. Gene expression levels were described as ratio between two absolute measurements (gene of interest/endogenous reference genes) to control for inter-sample variation. Before statistical analysis, all ratios were logarithmically transformed including a multiplier, which accounted the average Ct values obtained for each gene during the validation process. This procedure facilitated the comparison samples, which were run on different assay plates. Depending on the used genes and mutlipliers the inter-plate variation is around 5%.

### Statistical Analyses

Associations of gene expression levels and progression-free or overall survival were tested for each gene by the Kaplan-Meier method. Survival differences between the high and low expression group were analyzed by the log-rank test. To detect independent prognostic factors associated with overall and progression-free survival, multivariate Cox proportional hazards regression analysis with stepwise selection was applied. After adjustment for potential confounders, the following parameters were accounted for: pathological tumor stage (pT), lymph node involvement (pN), tumor grade (G) and the gene set. In addition, Receiver Operating Characteristic (ROC) curve analysis was performed to test the ability of the chosen cut-points to discriminate short survivors from long survivors [10], [11]. Recursive descent partition analysis was used to identify the strongest divisor of all factors and the most significant split determined by the largest likelihood-ratio chi-square statistic in relation to clinical response as described previously [12], [13]. The split was chosen to maximize the difference in the responses between the two branches of the split. The level of significance was set to P<0.05. All P values were based on two-sided tests. All statistical analyses were performed using the Software Packages Medcalc, Version 12.4.0 (Mariakerke, Belgium) and JMP 10.0 (SAS Institute, Cary, NC, USA).

The level of significance was set to p<0.05. All p values reported were based on two-sided tests. All statistical analyses were performed using the Software Packages SPSS® for Windows (Version 16.0, Chicago, Il, USA) and JMP 7.0 Software (SAS, Cary, NC, USA).

## Results

### Study group and tumor samples

Tissue blocks suitable for RNA extraction were retrieved from 47 patients and subjected to further analysis.

### Comparison of gene expression levels throughout subgroups

The gene expression levels of *EGFR* and *HPSE* showed a significant inverse correlation (p = 0.03). *FLT1* expression was correlated to *HPSE* expression (p<0.0001; Correlation Coefficient, CC = 0.74). Furthermore *FLT1* expression showed an inverse correlation to *PDGFA* expression (p = 0.006; CC = −0.55) and a positive correlation to the PDGFR expression (*PDGF-RA*; p = 0.0008; CC = 0.59). *HPSE* expression was also significantly associated with the expression of PDGFR-A (p<0.0001; CC = 0.78) but not to its substrate PDGF. The correlation of the other gene expression values are listed in Table 2.

**Table 2:** Spearman rank correlation between genes of interest.

		EGFR	FLT1	FLT4	HB-EGF	HIF1a	HPSE	PDGFA	PDGFRA	VEGF	VEGFC
	CC		−0.242	−0.243	−0.295	−0.015	−0.491	−0.307	−0.242	−0.307	0.189
EGFR	P		0,2915	0,2417	0,1821	0,9418	**0,0327**	0,1537	0,2657	0,1537	0,365
	n		21	25	22	25	19	23	23	23	25
	CC	−0.242		0.044	0.014	−0.268	0.735	−0.551	0.587	−0.024	−0.143
FLT1	P	0,2915		0,837	0,9503	0,1944	**<0.0001**	**0,0064**	**0,0008**	0,9101	0,5036
	n	21		24	22	25	27	23	29	24	24
	CC	−0.243	0.044		0.709	0.270	0.156	0.263	0.128	0.626	0.322
FLT4	P	0,2417	0,837		**<0.0001**	0,1109	0,487	0,1269	0,5079	**<0.0001**	0,0555
	n	25	24		38	36	22	35	29	39	36
	CC	−0.295	0.014	0.709		0.526	0.437	0.549	0.244	0.708	0.539
HB-EGF	P	0,1821	0,9503	**<0.0001**		**0,0014**	0,0615	**0,0008**	0,2288	**<0.0001**	**0,001**
	n	22	22	38		34	19	34	26	39	34
	CC	−0.015	−0.268	0.270	0.526		0.241	0.708	0.296	0.597	0.855
HIF1a	P	0,9418	0,1944	0,1109	**0,0014**		0,2797	**<0.0001**	0,1195	**0,0001**	**<0.0001**
	n	25	25	36	34		22	40	29	36	40
	CC	−0.491	0.735	0.156	0.437	0.241		−0.020	0.780	0.256	−0.100
HPSE	P	**0,0327**	**<0.0001**	0,487	0,0615	0,2797		0,9348	**<0.0001**	0,263	0,6581
	n	19	27	22	19	22		20	27	21	22
	CC	−0.307	−0.551	0.263	0.549	0.708	−0.020		0.182	0.466	0.678
PDGFA	P	0,1537	**0,0064**	0,1269	**0,0008**	**<0.0001**	0,9348		0,3638	**0,0048**	**<0.0001**
	n	23	23	35	34	40	20		27	35	39
	CC	−0.242	0.587	0.128	0.244	0.296	0.780	0.182		0.354	0.332
PDGF-RA	P	0,2657	**0,0008**	0,5079	0,2288	0,1195	**<0.0001**	0,3638		0,0645	0,0789
	n	23	29	29	26	29	27	27		28	29
	CC	−0.307	−0.024	0.626	0.708	0.597	0.256	0.466	0.354		0.580
VEGF	P	0,1537	0,9101	**<0.0001**	**<0.0001**	**0,0001**	0,263	**0,0048**	0,0645		**0,0003**
	n	23	24	39	39	36	21	35	28		35
	CC	0.189	−0.143	0.322	0.539	0.855	−0.100	0.678	0.332	0.580	
VEGFC	P	0,365	0,5036	0,0555	**0,001**	**<0.0001**	0,6581	**<0.0001**	0,0789	**0,0003**	
	n	25	24	36	34	40	22	39	29	35	

### Gene Expression and Survival

We used recursive decent partition tree analysis to find the factors showing the strongest association to survival and define the optimal cut-point of these factors. We used all available clinicopathological data and the measured genes for this model. Of the tested genes only EGFR, FLT1 and HPSE showed a correlation to survival in Spearman's test and the recursive decent partition tree analysis. Patients expressing *EGFR* above the 35^th^ percentile had a significantly worsened outcome (P = 0.04, hazard ratio [HR] = 2.84, 95% CI = 1.0959 to 7.3692; Figure 1) with a median overall survival of 8.5 months, whereas patients with lower *EGFR* expression had a median survival time of more than 3 years (38.5 months) as tested with Kaplan-Meier analysis. The same statistical test revealed that to the contrary patients with a higher *FLT1* expression had a higher chance for prolonged survival with a median overall survival time of 23.6 months and 40% of patients surviving longer than 3 years (P = 0.006, [HR] = 0.28, 95% CI = 0.07–1.14; Figure 2), whereas patients with a low expression of *FLT1* survived 5.3 months in median and none of the patients in this group survived longer than 2 years. Similar to *FLT1* patients with a high *HPSE* expression had a longer median survival time (P = 0.02, [HR] = 0.34, 95% CI = 0.11–1.04; Figure 3) with nearly one third of the patients living after 3 years, whereas none of the patients with a *HPSE* expression lower than the 35^th^ percentile reached this time point (median OS = 10.2 months).

**Figure 1:** Kaplan-Meier plot, estimating overall survival. Differences in survival between the high (interrupted line) and the low (continuous black line) *EGFR* expression group were analyzed with the log-rank test.

**Figure 2:** Kaplan-Meier plot, estimating overall survival. Differences in survival between the high (interrupted line) and the low (continuous black line) *FLT1* expression group were analyzed with the log-rank test.

**Figure 3:** Kaplan-Meier plot, estimating overall survival. Differences in survival between the high (interrupted line) and the low (continuous black line) *HPSE* expression group were analyzed with the log-rank test.

Only the genes with a significant (p<0.05) correlation to survival in univariate analysis (see above) were then put into a stepwise multivariate Cox proportional hazards regression model. In addition to *FLT1*, *HPSE*, *EGFR* mRNA expression clinical factors such as Age at Diagnosis, primary tumor expansion (pT), lymph node involvement (pN) and dedifferentiation grade were included in the model. The overall model fit had a significance level of p = 0.047. The factor that had the strongest significant independent association with survival-time in this patient cohort was low *FLT1* mRNA expression (20^th^ percentile cut-off) with a significance level of p = 0.04. Patients with a low *FLT1* expression had a nearly five times higher relative risk (4.74) of dying earlier.

### Receiver Operating Characteristic (ROC)

All three factors (expression of *FLT1*, *HPSE* and *EGFR*) were tested with ROC Analysis for their potential predictive capabilities in identifying patients with cholangiocarcinoma with a prolonged overall survival time (>3 years). The 35^th^ percentile cut-off of the *EGFR* mRNA expression showed 80% sensitivity (true positive rate) of and 75% specificity (true negative rate) for the diagnosis prolonged (>3 years) overall survival. The area under the curve was 0.775 (CI 0.583 to 0.908) with a significance level of p = 0.012. The positive likelihood ratio (true positive rate/false positive rate) was 3.2 and the negative likelihood ratio (false negative rate/true negative rate) 0.27. Both, *FLT1* and *HPSE*, were also significant when tested with the same criteria on ROC Curve Analysis, but with a specificity less than 40% (Figure 4).

**Figure 4:** Receiver Operating Characteristic (ROC) Curve Analysis for the potential of distinct EGFR expression to identify patients with risk of short vs. long (3–5 years) Survival.

## Discussion

We determined the gene expressions of *FLT1*, *FLT4*, *HPSE*, *Hif1a*, *HB-EGF*, *PDGFA*, *PDGF-RA* and *EGFR* in FFPE samples of patients with cholangiocarcinoma. By using laser capture microdissection to isolate tumor tissue from the clinical specimens along with quantitative RT-PCR, we hoped to achieve a more precise characterization of the associations of these gene expressions with each other and with patients' prognosis than was previously available. Of the chosen candidate genes three expression profiles seemed promising to be used in further studies, the fms-related tyrosine kinase 1 respectively vascular endothelial growth factor receptor 1 (*FLT1/VEGFR1*), heparanase (*HPSE*) and epidermal growth factor receptor (*EGFR*).

The latter gene has already been described and known to play a major role in tumorigenesis and aggressiveness of cancer, amongst others in lung cancer. Recent publications evaluated the role of anti-*EGFR* therapies in biliary tracts carcinomas. Chiorean and colleagues tested Erlotinib and Docetaxel in Advanced and Refractory Hepatocellular and Biliary Cancers in a Phase II Trial of the Hoosier Oncology Group GI06-101 [14]. They came to the conclusion that anti-EGFR therapy remains to be an important possibility in these tumors but only with a molecular “targeted” approach. We were able to show that a high *EGFR* mRNA expression level (>35th percentile) is associated to patients' survival and confers a significantly worsened chance to survive longer than one year (P = 0.04, hazard ratio [HR] = 2.84), whereas patients with lower *EGFR* expression had a median survival time of more than 3 years (38.5 months). These results are in agreement with conclusions from other groups [15] that also indicated a higher chance for better outcome in low expression groups. With receiver operating characteristic (ROC) curve analysis we were able to show that the 35th percentile cut-off of the *EGFR* mRNA expression could be useful in identifying those patients at risk for shortened survival with a sensitivity (true positive rate) of 80% and a specificity (true negative rate) of 75%. As Andersen and colleagues recently published the selection of patients from high risk groups may indicate the necessity of modified treatment and seems to be useful also in cholangiocarcinoma [16].

It has already been discussed by other groups that measuring genes from the angiogenesis pathway seems to be a promising approach in tumors of the biliary tract and pancreas, especially due to their hypoxic nature [17]. In preceding works we were able to shed light on a strong association of *Hif1a* expression with survival in pancreatic cancer and soft tissue sarcomas [4], [5]. However, this association was not significant in the examined study group of patients with cholangiocarcinoma which is in concordance with discoveries from other groups examining *Hif1a* in CCC [18] who were also not able to show a correlation of *Hif1a* expression to survival.

*VEGFR 2/3* expression was tested in several studies so far [19]. There is however only limited data available for the expression of *FLT1*/*VEGFR1* in cholangiocarcinoma though Rogler and others suggested a potential association with a more aggressive phenotype [20]. We were able to show for the first time that *FLT1* seems to be independently associated with overall survival of patients with a biliary tract tumor. Interestingly Kaplan-Meier Analysis revealed that patients with a higher *FLT1* expression potentially have a better outcome, though one would anticipate high expression to indicate a more aggressive tumor. Patients with a high expression showed a median overall survival time of 23.6 months and 40% of patients surviving longer than 3 years (P = 0.006, [HR] = 0.28). The independent association of high *FLT1* expression with better outcome was supported by a stepwise multivariate Cox proportional hazards regression model. In this study group *FLT1* was the strongest independent factor associated with overall survival.

Especially due to the destructive locally invasive behavior and a high rate of distant metastasis we already tested *HPSE* in pancreatic cancer [21]. Although we were not able to affirm a significant correlation to overall survival we revealed the link of *HPSE* expression to a higher rate of lymph node invasion, hence a more aggressive tumor type. In this study we were able to show that similar to *FLT1* none of the patients with a *HPSE* expression lower than the 35^th^ percentile reached the 2-year mark (median OS = 10.2 months). Although *FLT1* and *HPSE* proved to be significantly linked with overall survival they were - in contrast to *EGFR* - not usable to distinguish patients at high risk for worsened overall survival with sufficient sensitivity and specificity – at least not in the examined study group. This may be explainable by the size of the study group or may indicate that although *FLT1* and *HPSE* are potential markers to predict outcome they are not usable as such as stand-alone markers, which may explain the discordant findings in relation to other studies. Interestingly the dichotomized (cut-point) *FLT1* mRNA expression showed a significant but inverse correlation to the pathological tumor stage (p = 0.001; Table 3).

**Table 3:** Spearman rank correlation between clinicopathological characteristics and dichotomized expression values.

		Age	Gender	Grading	pN	pT	EGFR Split	FLT1 Split	HPSE Split
	CC		−0,248	−0,205	−0,292	0,078	0,009	−0,315	−0,089
Age	P		0,0933	0,1766	0,2402	0,6074	0,9643	0,09	0,6592
	n		47	45	18	46	29	30	27
	CC	−0,248		0,086	0,158	−0,047	−0,099	0,017	−0,246
Gender	P	0,0933		0,5754	0,5309	0,7567	0,608	0,9281	0,2155
	n	47		45	18	46	29	30	27
	CC	−0,205	0,086		0,553	0,082	0,345	−0,022	−0,098
Grading	P	0,1766	0,5754		**0,0172**	0,5942	0,0722	0,9084	0,6353
	n	45	45		18	45	28	29	26
	CC	−0,292	0,158	0,553		0,012	0,501	0,051	−0,267
pN	P	0,2402	0,5309	**0,0172**		0,9631	0,0814	0,8675	0,428
	n	18	18	18		18	13	13	11
	CC	0,078	−0,047	0,082	0,012		0,107	−0,572	−0,258
pT	P	0,6074	0,7567	0,5942	0,9631		0,5896	**0,0012**	0,2024
	n n	46	46	45	18		28	29	26
EGFR	CC	0,009	−0,099	0,345	0,501	0,107		−0,208	−0,519
Split	P	0,9643	0,608	0,0722	0,0814	0,5896		0,3649	**0,0228**
	n	29	29	28	13	28		21	19
FLT1	CC	−0,315	0,017	−0,022	0,051	−0,572	−0,208		0,596
Split	P	0,09	0,9281	0,9084	0,8675	**0,0012**	0,3649		**0,001**
	n	30	30	29	13	29	21		27
HPSE	CC	−0,089	−0,246	−0,098	−0,267	−0,258	−0,519	0,596	
Split	P	0,6592	0,2155	0,6353	0,428	0,2024	**0,0228**	**0,001**	
	n	27	27	26	11	26	19	27	

It should be pointed out that our present study has been retrospectively conducted in samples collected from patients that were treated consecutively in our clinic. Accordingly, the results may have been influenced by confounders that have occurred during the follow-up period but were not reported, and by additional bias [22]. Studies like the one we conducted may therefore not be used to directly be translated into clinical practice but may help understand a tumor that until now defies classical unselected treatment approaches. The results have to be validated in prospectively collected study groups. Nonetheless - as discussed before - identifying genes that are associated with an aggravated outcome is an important method to form a candidate oncogene pool that is available for further work, such as in vitro studies or biomarker guided therapy trials [4]. Further studies are warranted and currently employed by our group to validate these genes including tactics to identify these genes in circulating tumor cells [23], [24].

## Conclusions

The significant association of high *EGFR* expression on survival probability and the high sensitivity and specificity of measuring *EGFR* expression to identify patients at risk for a shorter survival suggests that *EGFR* may be a useful candidate for treatment selection in cholangiocarcinomas. Furthermore *FLT1* was independently associated with survival in our study group and stronger associated with outcome than other clinicopathologic parameters. The significant associations of *EGFR*, *FLT1* and *HPSE* gene expression with survival warrant prospective evaluation of their usability in selecting more efficient treatment strategies for patients with cholangiocarcinoma.
